The article "Peitu Shengjin Recipe Attenuates Airway Inflammation via the TLR4/NF-kB Signaling Pathway on Chronic Obstructive Pulmonary Disease" was published in 2022. Journal: Evid Based Complement Alternat Med.

# Peitu Shengjin Recipe Attenuates Airway Inflammation via the TLR4/NF-kB Signaling Pathway on Chronic Obstructive Pulmonary Disease

**DOI:** 10.1155/2022/2090478

**Published:** 2022-08-12

**Authors:** Xuzhen Hu, Bo Hong, Minghuan Sun

**Affiliations:** Respiratory Department, Ningbo City Hospital of Traditional Chinese Medicine, Ningbo, Zhejiang 315000, China

## Abstract

**Background:**

Chronic obstructive pulmonary disease (COPD) is a common respiratory disease, but there is no specific medicine for COPD. In this study, we aimed to evaluate the effects of Peitu Shengjin Recipe (PSR) and Biostime Probiotic Powder on COPD rats.

**Methods:**

UPLC-Q/TOF-MS was used to detect the chemical constituents in PSR. The COPD rat model was established by cigarette smoke combined with tracheal injection of lipopolysaccharide. We assessed lung function by calculating FEV_0.3_/FVC%, dynamic lung compliance (Cdyn), and resistance of inspiration (RI). Histological analysis was performed by HE staining. The levels of TNF-*α,* IFN-*γ*, IL-1*β*, IL-4, and IL-10 were detected by the ELISA. The mRNA and protein expressions of the TLR4/NF-kB signaling pathway were detected by the qRT-PCR and western blotting, respectively.

**Results:**

There were 53 ESI^+^ and 50 ESI^−^ components in PSR. After high-dose PSR treatment, FEV_0.3_/FVC% and Cdyn increased significantly, while RI decreased. Compared with the COPD model, the RI of the Biostime Probiotic Powder group was significantly lower. HE staining showed that the inflammatory cell infiltration was reduced to varying degrees, the bronchial tube wall was not thickened, and the alveoli were relatively intact after treatment with PSR and Biostime Probiotic Powder. Compared with the model group, the levels of TNF-*α*, IFN-*γ*, IL-1*β*, IL-4, and IL-10 in the PSR group and the Biostime Probiotic Powder group were reversed. The mRNA and protein expressions of TLR4 and NF-kB were significantly decreased after PSR and Biostime Probiotic Powder treatment.

**Conclusion:**

Our findings suggest that PSR and Biostime Probiotic Powder have protective effects on COPD rats, which may be achieved by modulating the TLR4/NF-kB signaling pathway.

## 1. Introduction

Chronic obstructive pulmonary disease (COPD) is one of the leading causes of morbidity and mortality, characterized by persistent airflow limitation and increased chronic inflammatory response in lung tissue [1, 2]. It is widely accepted that the primary mechanism of COPD is chronic inflammation, including the release of inflammatory cytokines and immune cell responses [3]. Cigarette smoke and intratracheal administration of lipopolysaccharide (LPS) to rats are considered an ideal model of COPD. Previous studies have shown that cigarette smoke and LPS can stimulate airway epithelial cells to release harmful molecules that bind to toll-like receptor 4 (TLR4) on the cell surface [4, 5]. Activation of TLR4 induces nuclear factor kappa B (NF-kB) and inflammatory cytokines, such as tumor necrosis factor alpha (TNF-*α*) [6, 7] and interleukin-1 beta(IL-1*β*) [8–10]. Therefore, the TLR4/NF-kB signaling pathway may play an important role in the pathogenesis of COPD.

The article "Peitu Shengjin Recipe Attenuates Airway Inflammation via the TLR4/NF-kB Signaling Pathway on Chronic Obstructive Pulmonary Disease" was published in 2022. Journal: Evid Based Complement Alternat Med.

It is reported that Chinese medicine has prominent advantages in the prevention and treatment of chronic diseases [11–18]. Peitu Shengjin Recipe (PSR) is a traditional Chinese herbal compound that varies slightly according to the patient's condition or individual differences. It has been reported that traditional Chinese medicine may be an alternative treatment method for COPD patients [19–21]. For example, BuzhongYiqi Decoction could improve lung function and sports ability [22], and Feikang granules could ameliorate pulmonary inflammation in COPD rats by the TLR2/4 mediated NF-kB pathway [4]. Gong et al. reported that PSR could improve nutritional status and immune function in stable phase COPD patients [23]. In addition, the intestinal probiotics of COPD patients were significantly lower than that of healthy people [24]. Biostime Probiotic Powder has various functions, including promoting probiotic proliferation, inhibiting pathogenic bacteria, and enhancing metabolism and immune function [25, 26]. However, the effect and mechanism of Biostime Probiotic Powder on COPD have not been clearly studied.

In this study, we established a COPD rat model by exposure to cigarette smoke and intratracheal administration of LPS. PSR and Biostime Probiotic Powder were used to treat COPD rats. The effects of PSR and Biostime Probiotic Powder on COPD rats were evaluated by HE staining, ELISA, qRT-PCR, and western blotting.

## 2. Materials and Methods

### 2.1. Reagents

Paraxylene, absolute alcohol, citrate buffer, and phosphate buffer were purchased from SINOPHARM (Beijing, China). The enzyme-linked immunosorbent assay (ELISA) kits for TNF-*α*, IFN-*γ,* IL-1*β,* IL-4, and IL-10 were purchased from R&D Systems (Minneapolis, USA). The SYBR Green qPCR kit and reverse transcription kit were purchased from CWBIO (Beijing, China). The BCA protein assay kit and chemiluminescence detection reagent were purchased from Solarbio (Beijing, China). Anti-TLR4/MD2 complex (ab95562) and anti-NF-*κ*B p65 (ab207297) were purchased from Abcam (Cambridge, USA). PSR decoction was prepared by the Ningbo City Hospital of Traditional Chinese Medicine. Biostime Probiotic Powder was purchased from BIOSTIME (Guangzhou, China).

The article "Peitu Shengjin Recipe Attenuates Airway Inflammation via the TLR4/NF-kB Signaling Pathway on Chronic Obstructive Pulmonary Disease" was published in 2022. Journal: Evid Based Complement Alternat Med.

### 2.2. UPLC-Q/TOF-MS Analysis

Chromatographic analysis was conducted on the Waters ACQUITY I-Class Plus UPLC system (Waters Corp., Milford, USA) and ACQUITY UPLC BEH C18 (100 × 2.1 mm, 1.7 *μ*m, AB SCIEX, Framingham, USA). The mobile phase was a mixture of acetonitrile with 0.1% formic acid and water with 0.1% formic acid. The gradient elution conditions were as follows: 0–2 min, 99% B; 2–12 min, 99%–55% B; 12～19 min, 55%–1% B. MS spectrometry was performed on the SCIEX X-500R quadrupole time of flight mass spectrometer (AB SCIEX, Framingham, USA). The parameters were set as follows: ion source gas1 (Gas1):45, ion source gas2 (Gas2):55, curtain gas (CUR):35, source temperature: 600°C, ionSapary voltage floating (ISVF):5500 V/−4500 V; TOF MS scan m/z range:100–1500 Da, production scan m/z range:25–1500 Da, TOF MS scan accumulation time: 0.25 s/spectra, and product ion scan accumulation time: 0.035 s/spectra. SCIEX OS software was used to collect and analyze data.

### 2.3. Animal and Group

Thirty male Sprague-Dawley (SD) rats, weighing 200 ± 20 g, were purchased from the Zhejiang Medical Laboratory Animal Center (Hangzhou, China). Fifty-five rats were randomly selected to replicate the COPD model through cigarette smoke combined with LPS. Rats were treated with 200 *μ*l LPS (1 mg/ml) by gavage on days 1 and 14. From day 2 to day 28, rats were placed in a box and exposed to the smoke produced by a lighted cigarette for one hour per day. Carbon dioxide asphyxiation was performed before rats were dissected. The rats were divided into six groups: control group, model group, low, medium, and high-dose of the PSR group, and Biostime Probiotic Powder group. According to the dose conversion between adults and rats, the PSR-medium dose group was given 1.5 times the low dose, and the high-dose group was given three times the low dose. The rats in the normal group and the model group were given an equal volume of normal saline by oral gavage. Biostime Probiotic Powder was converted to rat dosage by gavage according to the instructions. All experiments were approved by the Animal Ethics Committee (EYOUNG-20201117-06), and this study was conducted in accordance with the National Institute of Health's Guideline for the Care and Use of Laboratory Animals.

### 2.4. Lung Function Assessment and HE Staining

After the last administration, lung function was measured by using an animal lung function analysis system (AniRes2005, Beijing, China). Rats were anesthetized, tracheostomized, and then connected to the instrument. FEV_0.3_/FVC%, dynamic lung compliance (Cdyn), and resistance of inspiration (RI) were tested. Lung tissue was fixed with 4% paraformaldehyde and embedded in paraffin. Then, we used hematoxylin-eosin (HE) to stain sections (4 *μ*m thick). The light microscope was used to observe it.

The article "Peitu Shengjin Recipe Attenuates Airway Inflammation via the TLR4/NF-kB Signaling Pathway on Chronic Obstructive Pulmonary Disease" was published in 2022. Journal: Evid Based Complement Alternat Med.

### 2.5. ELISA

Blood samples were collected from the abdominal aorta and centrifuged at 3000 rpm/min for 15 min. According to the manufacturer's instructions, the levels of TNF-*α*, IFN-*γ*, IL-1*β*, IL-4, and IL-10 in the supernatant were determined using the ELISA kits (MEIMIAN, Jiangsu, China). The details of the ELISA were as follows: (1) We prepare and dilute reagents. (2) We set standard, sample, and control wells. 100 *μ*l of the horseradish peroxidase-labeled antibody was added to the standard and sample wells. (3) The plate was incubated in a 37°C water bath for 60 min. (4) After washing, the chromogenic reagent was added to the plate for 15 min at 37°C. (5) The absorbance value was measured at 450 nm.

### 2.6. qRT-PCR

Total RNA was extracted from lung tissue with the Trizol reagent and reverse transcribed into cDNA. The reaction conditions were as follows: 15 min at 42°C and 5 min at 85°C. qRT-PCR was detected using the LightCycler ® 96 instrument (Roche, Basel, Switzerland), and the reaction conditions were as follows: denaturation at 95°C for 10 min; 15 s at 95°C; 60 s at 60°C (40 cycles). The primers were as follows: TLR4 (forward, AACTCTGCGCCTAAAACCCA, reverse, TGCTACTTCCTTGTGCCCTG), NF-*κ*B (forward, ACAGATTCTGGGGAGTGTGC, reverse, GAGCCGACTATCGTACAGGG), and GAPDH (forward, GATGGTGAAGGTCGGTGTGA, reverse, TGAACTTGCCGTGGGTAGAG).

### 2.7. Western Blotting

Lung tissues were homogenized with lysis buffer and centrifuged at 4°C for 5 min, and the supernatant was taken. The total protein concentration of the samples was assayed using the BCA kits (Solarbio, Beijing, China). Samples were separated on 5% SDS-PAGE, transferred to PVDF membranes (GE Healthcare Life, Atlanta, USA), and blocked with 5% skim milk for 1.5 h. After 3 washes with TBST, the membrane was incubated overnight at 4°C with primary antibodies, including anti-TLR4/MD2 complex, anti-NF-*κ*B p65, and anti-GAPDH (HUABIO, Hangzhou, China). Then, the membrane was washed with TBST three times. We incubated the membrane for 2 hours at room temperature using the appropriate horseradish peroxidase-conjugated secondary antibody. The enhanced chemiluminescence kit (Solarbio, Beijing, China) was utilized to visualize the membrane. At last, we used ImageJ software to calculate the relative protein levels.

### 2.8. Statistical Analysis

All values were expressed as the mean ± SD. GraphPad Prism software (Version 7.0, San Diego, USA) was used for statistical comparisons. The *P* value < 0.05 was regarded as statistically significant. For pairwise comparison between the groups, two independent samples *t*-test was used for homogeneous variances, and the Kruskal–Wallis H test was used for unequal variances.

The article "Peitu Shengjin Recipe Attenuates Airway Inflammation via the TLR4/NF-kB Signaling Pathway on Chronic Obstructive Pulmonary Disease" was published in 2022. Journal: Evid Based Complement Alternat Med.

## 3. Results

### 3.1. Components of Peitu Shengjin Recipe

The chemical composition of PSR was analyzed by UPLC-Q/TOF-MS in positive and negative ESI detection modes. The total ion flow diagram of PSR is shown in Figure 1. 53 and 50 components of PSR were identified by the positive and negative ion mode, respectively. It included amino acids, alkaloids, volatile oils, fatty acids, and other components, as given in Table 1 and Table 2.

### 3.2. Effects of Peitu Shengjin Recipe and Biostime Probiotic Powder on Lung Function

As shown in Table 3 and Figure 2, we measured FEV_0.3_/FVC%, Cdyn, and RI to show the effect of PSR and Biostime Probiotic Powder on lung function. Compared with the controls, FEV_0.3_/FVC% and Cdyn were significantly decreased, whereas RI was enhanced in the model group. After treatment of PSR and Biostime Probiotic Powder, there was no significant difference of FEV_0.3_/FVC%, Cdyn, and RI in the PSR-low dose group and the PSR-medium dose group (*P* > 0.05). FEV_0.3_/FVC% and Cdyn increased (*P* < 0.05), and RI significantly decreased (*P* < 0.01) in the PSR-high dose group. There were no remarkable changes in FEV_0.3_/FVC% and Cdyn, but RI values in the Biostime Probiotic Powder group were statistically different. In addition, we stained lung tissues of the six groups with HE (Table 4 and Figure 3). In the controls, the bronchus was intact and the mucosa was not shedding, and there was no inflammatory cell infiltration. In the model group, the bronchus was broken incompletely, the trachea was shrunk, the lumen was narrowed, the tracheal mucosa was detached, and a large number of inflammatory cells were infiltrated around. The tracheal mucosa was intact in the low, medium, and high-dose groups of PSR, and the peripheral inflammatory cell infiltration was less than that in the model group. The Biostime Probiotic Powder group also had a protective effect on lung tissue.

### 3.3. Effects of Peitu Shengjin Recipe and Biostime Probiotic Powder on Inflammatory Factors

TNF-*α*, IFN-*γ*, IL-1*β*, IL-4, and IL-10 in serum were measured by the ELISA. As shown in Figure 4, the serum levels of TNF-*α*, IFN-*γ*, and IL-1*β* in the model group were significantly higher than those in the control group, and IL-4 and IL-10 levels were significantly decreased (*P* < 0.01). Compared with the model group, IFN-*γ* levels obviously decreased in the PSR-low dose group; TNF-*α* and IFN-*γ* levels significantly decreased in the PSR-medium dose group; the serum levels of TNF-*α*, IFN-*γ*, and IL-1*β* significantly decreased in the PSR-high dose group, whereas IL-4 and IL-10 increased (*P* < 0.01). In the Biostime Probiotic Powder group, the levels of TNF-*α* and IFN-*γ* were decreased, the levels of IL-4 were increased, and the levels of IL-1*β* and IL-10 had no significant changes.

The article "Peitu Shengjin Recipe Attenuates Airway Inflammation via the TLR4/NF-kB Signaling Pathway on Chronic Obstructive Pulmonary Disease" was published in 2022. Journal: Evid Based Complement Alternat Med.

### 3.4. Effects on Peitu Shengjin Recipe and Biostime Probiotic Powder on the TLR4/NF-kB Pathway

Figure 5(a) shows that the mRNA level of TLR4 in the PSR-high dose group was significantly decreased compared with that of the COPD model group. After treatment with high-dose PSR and Biostime Probiotic Powder, NF-kB expression was significantly increased (*P* < 0.05). Meanwhile, we performed the western blotting to detect the protein levels of TLR4 and NF-kB p65 (Figure 5(b)). The results showed that the expression level of TLR4 protein in the PSR-medium dose group was significantly decreased (*P* < 0.05). The levels of TLR4 and NF-kB p65 in the lung tissue of rats in the PSR-medium dose group and the Biostime Probiotic Powder group were significantly decreased (*P* < 0.01).

## 4. Discussion

In this study, we identified the chemical composition of PSR. The therapeutic effects of PSR and Biostime Probiotic Powder on COPD rats were also explored. Our results showed that PSR and Biostime Probiotic Powder attenuated airway inflammation in COPD rats by downregulating the TLR4/NF-kB signaling pathway.

COPD will be the third leading cause of death by 2030 [27]. The current pharmacological treatments include bronchodilators and antibiotics combined with corticosteroids, which could not cure COPD [28, 29]. Inhibition of TLRs has been reported to be a key cellular target for initiating and sustaining inflammation and improving lung function and thus playing a therapeutic role in COPD patients [30]. TLR4 is the first identified mammalian TLR, expressed in inflammatory cells. In lung tissue, TLR4 may be activated by risk factors such as smoking, inhalation of contaminated air, and bacterial and viral infections, which in turn activate NF-kB and induce the expression of inflammatory mediators [31]. In the study, we established the COPD model in rats by combining smoking and LPS. The results of lung function assessment and HE staining showed the damages of lung tissue in COPD rats. In addition, the ELISA assay indicated that the COPD model induced the release of TNF-*α*, IFN-*γ*, and IL-1*β* and decreased levels of IL-4 and IL-10. This finding is consistent with a previous research study. Alexander et al. observed an increase of TNF-*α* and IL-1*β* in bronchoalveolar lavage of long-term smokers [32]. Wang et al. reported that LPS enhanced the expression of IFN-*γ* in rat pulmonary artery smooth muscle cells through the TLR4/IRAK/NF-kB pathway [31]. Moreover, Gu et al. showed a significant decrease in serum IL-4 and IL-10 concentrations [33].

The article "Peitu Shengjin Recipe Attenuates Airway Inflammation via the TLR4/NF-kB Signaling Pathway on Chronic Obstructive Pulmonary Disease" was published in 2022. Journal: Evid Based Complement Alternat Med.

Medicinal plants have been reported to have many biological effects [34–41]. In China, PSR has been shown to have clinical efficacy in the treatment of COPD patients [23, 42, 43]. PSR is composed of Astragalus, Codonopsis, Angelica, Atractylodes, Fructus aurantii, peach kernel, tangerine peel, Poria cocos, Pinellia ginger, Platycodon grandiflorum, and licorice [44]. PSR has the effect of invigorating the spleen and nourishing the lung. Our results showed that the components of PSR included nobiletin, isoliquiritigenin, 7-hydroxycoumarin, caffeic acid, and so on. Nobiletin has been reported to exhibit anti-inflammatory, anticancer, and anti-insulin resistance activities. Li et al. found that nobiletin has a protective effect on lung injury by inhibiting NF-kB activation [22]. Isoliquiritigenin also possesses antioxidative and anti-inflammatory properties by inhibiting the NF-kB and NLRP3 pathways [23]. Jose et al. found that 7-hydroxycoumarin has effects on the apoptosis and the cell cycle of human lung cancer cells [23]. Meanwhile, caffeic acid was found to have anti-inflammatory and ameliorative effects against tobacco smoking on the lung, heart, and kidney [45]. The underlying mechanism of PSR on COPD might be related to nobiletin, isoliquiritigenin, and other components. Therefore, we explored the mechanisms of different doses of PSR in COPD rats. The ELISA showed that PSR significantly affected the levels of TNF-*α*, IFN-*γ*, IL-1*β*, IL-4, and IL-10 in a dose-dependent manner. In the TLR4/NF-kB signaling pathway, high-dose PSR could significantly downregulate the expression of TLR4 and NF-kB. This suggests PSR may improve inflammatory status in the lung, and the effect is dose-dependent. It provided a theoretical basis for further clinical application of PSR. At the same time, we assessed the effects of Biostime Probiotic Powder on COPD rats. It also has a therapeutic effect on COPD but is not superior to high-dose PSR. The results indicated that Biostime Probiotic Powder significantly decreased the levels of TNF-*α* and IFN-*γ* and increased the concentration of IL-4 in serum. The western blotting and qRT-PCR showed that Biostime Probiotic Powder significantly reduced the expression of NF-kB. It is suggested that Biostime Probiotic Powder could play a vital role in the treatment of COPD by regulating inflammatory cytokines through the TLR4/NF-kB signaling pathway. In clinic, Biostime Probiotic Powder might be used to cure COPD.

In conclusion, our results demonstrated that PSR and Biostime Probiotic Powder had a protective effect against COPD. PSR and Biostime Probiotic Powder could improve lung function, reverse the levels of inflammation-related cytokines, and regulate the mRNA and protein expressions of the TLR4/NF-kB signaling pathway. The therapeutic effect of PSR and Biostime Probiotic Powder was attributed to the inhabitation of the TLR4/NF-kB signaling pathway. Hence, our study showed that PSR and Biostime Probiotic Powder are promising therapeutic targets for COPD.

The article "Peitu Shengjin Recipe Attenuates Airway Inflammation via the TLR4/NF-kB Signaling Pathway on Chronic Obstructive Pulmonary Disease" was published in 2022. Journal: Evid Based Complement Alternat Med.

## Figures and Tables

**Figure 1:** The total ion flow diagram of Peitu Shengjin Recipe by UPLC-Q/TOF-MS. (a) Positive mode. (b) Negative mode.

**Figure 2:** Peitu Shengjin Recipe and Biostime Probiotic Powder improved the lung function of rats with COPD. (a) FEV0.3/FVC (%). (b) Dynamic lung compliance (Cdyn). (c) Resistance of inspiration (RI). *Note*: ^▲^*P* < 0.05 and ^▲▲^*P* < 0.01 vs. the control group; ^★^*P* < 0.05 and ^★★^*P* < 0.01 vs. the model group.

**Figure 3:** The effects of Peitu Shengjin Recipe and Biostime Probiotic Powder on lung tissue. (a) Control group. (b) Model group. (c) PSR-low dose group. (d) PSR-medium dose group. (e) PSR-high dose group. (f) Biostime Probiotic Powder group.

**Figure 4:** Serum levels of TNF-*α*, IFN-*γ*, IL-1*β*, IL-4, and IL-10 in rats. *Note*: ^▲^*P* < 0.05 and ^▲▲^*P* < 0.01 vs. the control group; *P* < 0.05 and *P* < 0.01 vs. the model group.

**Figure 5:** The expressions of TLR4 and NF-kB p65 in lung tissue. (a) mRNA levels; (b) protein levels. *Note*: ^▲^*P* < 0.05 and ^▲▲^*P* < 0.01 vs. the control group; *P* < 0.05 and *P* < 0.01 vs. the model group.

**Table 1:** The chemical components of Peitu Shengjin Recipe in the positive mode.

NO.	Component name	Area	Retention time	Formula	Precursor mass	Found at mass	Mass error (ppm)	Library score	Isotope ratio difference
1	Histidine	1.98*E* + 05	1.39	C_6_H_9_N_3_O_2_	156.077	156.0768	0.5	95.4	0.7
2	L(+)-Arginine	8.20*E* + 06	1.4	C_6_H_14_N_4_O_2_	175.119	175.1188	−1.1	80	0.9
3	Threonine	3.61*E* + 05	1.47	C_4_H_9_NO_3_	120.066	120.0654	−1.0	86.6	1.1
4	Glutamic acid	4.45*E* + 05	1.51	C_5_H_9_NO_4_	148.06	148.0604	−0.3	96.9	0.7
5	Betaine	5.75*E* + 05	1.52	C_5_H_11_NO_2_	118.086	118.0862	−0.4	100	0.1
6	Sorbitol	3.08*E* + 05	1.53	C_6_H_14_O_6_	183.086	183.0863	0	93.3	0.6
7	Trigonelline	1.51*E* + 06	1.59	C_7_H_7_NO_2_	138.055	138.0547	−1.9	95.9	0.8
8	Proline	4.67*E* + 06	1.62	C_5_H_9_NO_2_	116.071	116.0704	−1.9	99.2	0.8
10	Adenine	7.04*E* + 05	1.67	C_5_H_5_N_5_	136.062	136.0616	−1.1	89	1.8
9	Stachydrine	9.68*E* + 06	1.67	C_7_H_13_NO_2_	144.102	144.1016	−1.8	100	0.2
11	Nicotinic acid	2.74*E* + 05	2.36	C_6_H_5_NO_2_	124.039	124.0393	−0.3	95.4	0.2
12	Nicotinamide	1.66*E* + 05	2.52	C_6_H_6_N_2_O	123.055	123.0552	−0.5	97.8	1.7
13	6-Hydroxypurine	8.76*E* + 04	2.66	C_5_H_4_N_4_O	137.046	137.0458	−0.3	75	1
14	Adenosine	1.16*E* + 06	4.95	C_10_H_13_N_5_O_4_	268.104	268.1038	−0.7	100	0.9
15	Guanosine	2.38*E* + 05	5.18	C_10_H_13_N_5_O_5_	284.099	284.0992	1.0	100	0.8
16	Phenylalanine	6.42*E* + 05	6.09	C_9_H_11_NO_2_	166.086	166.0862	−0.6	98.3	1.1
17	Esculin hydrate	3.71*E* + 04	7.84	C_15_H_16_O_9_	341.087	341.0874	2.1	75.5	1.3
18	Chlorogenic acid	1.59*E* + 05	8.39	C_16_H_18_O_9_	355.102	355.1025	0.5	99.1	1.1
19	Cryptochlorogenic acid	1.59*E* + 05	8.39	C_16_H_18_O_9_	355.102	355.1025	0.5	99.1	1.1
20	Typhaneoside	2.48*E* + 04	9.43	C_34_H_42_O_2_0	771.234	771.2348	0.7	78.8	3
21	Schaftoside	2.67*E* + 05	9.58	C_26_H_28_O_14_	565.155	565.1557	1.0	97.6	2.3
22	Calycosin-7-O-glucoside	2.54*E* + 06	10.45	C_22_H_22_O_10_	447.129	447.1283	−0.5	100	0.3
23	Eriodictyol	5.46*E* + 05	10.59	C_15_H_12_O_6_	289.071	289.0707	0.2	93.4	1.3
24	PolygalaxanthoneIV	6.77*E* + 05	10.59	C_27_H_32_O_15_	597.181	597.1818	0.6	90.8	2.4
25	Isoliquiritigenin	3.94*E* + 06	10.67	C_15_H_12_O_4_	257.081	257.0806	−1.0	92.2	0.7
26	7-Hydroxycoumarin	3.82*E* + 05	10.85	C_9_H_6_O_3_	163.039	163.0389	−0.2	86.5	0.2
27	Isoferulic acid	2.11*E* + 05	10.9	C_10_H_10_O_4_	195.065	195.0651	−0.4	97.2	1.2
28	Naringenin	9.48*E* + 06	11.3	C_15_H_12_O_5_	273.076	273.0757	−0.2	100	0.5
29	Narirutin	9.62*E* + 06	11.3	C_27_H_32_O_14_	581.186	581.1867	0.4	90.3	3.6
30	Hesperetin	7.56*E* + 06	11.7	C_16_H_14_O_6_	303.086	303.0864	0.3	100	1.4
31	Hesperidin	1.08*E* + 07	11.7	C_28_H_34_O_15_	611.197	611.197	0	92.2	1.3
32	Apigenin 7-O-beta-D-glucuronide	6.53*E* + 04	12.35	C_21_H_18_O_11_	447.092	447.093	1.8	95	0.5
33	Ononin	1.81*E* + 06	12.47	C_22_H_22_O_9_	431.134	431.134	0.8	98.6	0.5
34	Methylhesperidin	5.94*E* + 04	12.48	C_29_H_36_O_15_	625.213	625.2127	0	93.9	4.7
35	6,7-Dimethoxycoumarin	5.10*E* + 04	12.51	C_11_H_10_O_4_	207.065	207.0652	0.2	87.8	2.5
36	Isomucronulatol	9.71*E* + 04	13.11	C_17_H_18_O_5_	303.123	303.1229	0.6	96.5	1.7
37	Xanthotoxol	1.38*E* + 05	13.32	C_11_H_6_O_4_	203.034	203.034	0.3	76.3	2.1
38	Wogonin 7-O-glucuronide	2.61*E* + 04	13.52	C_22_H_20_O_11_	461.108	461.1083	1.1	100	4.2
39	Tectorigenin	1.12*E* + 05	14.02	C_16_H_12_O_6_	301.071	301.0707	0	82.1	0.1
40	AstragalosideIV	1.07*E* + 05	14.68	C_41_H_68_O_14_	785.468	785.4687	0.7	92.3	3.2
41	Glycyrrhizic acid	9.83*E* + 06	14.85	CVH_62_O_16_	823.411	823.4109	−0.2	96.7	3.7
42	Formononetin	1.31*E* + 06	15.1	C_16_H_12_O_4_	269.081	269.0806	−1.0	99.6	0.9
43	Limonin	6.50*E* + 06	15.48	C_26_H_30_O_8_	471.201	471.2015	0.4	91.4	1.6
44	Isovanillin	7.98*E* + 04	15.51	C_8_H_8_O_3_	153.055	153.0546	0	92.1	1.3
45	Nobiletin	4.66*E* + 07	15.82	C_21_H_22_O_8_	403.139	403.1382	−1.4	98	0.5
46	Tangeretin	3.52*E* + 07	16.39	C_20_H_20_O_7_	373.128	373.1276	−1.5	98.4	0.2
47	Parthenolide	5.82*E* + 04	16.56	C_15_H_20_O_3_	249.149	249.1485	−0.2	80.6	2
48	3-N-butyl-4,5-dihydrophthalide	8.80*E* + 04	16.56	C_12_H_16_O_2_	193.122	193.1222	−0.8	90.7	2
49	Glabridin	2.34*E* + 04	17.04	C_20_H_20_O_4_	325.143	325.1437	0.7	97.8	3.1
50	Osthole	9.77*E* + 04	17.33	C_15_H_16_O_3_	245.117	245.1172	0.1	91.7	1.1
51	Anisaldehyde	1.76*E* + 05	17.59	C_8_H_8_O_2_	137.06	137.0596	-0.8	95.4	0.5
52	Isoalantolactone	1.57*E* + 05	17.65	C_15_H_20_O_2_	233.154	233.1537	0.3	95.6	1.7
53	Patchouli alcohol (loss H_2_0)	1.26*E* + 04	19.31	C_15_H_24_	205.195	205.195	−0.5	90.7	1.7

The article "Peitu Shengjin Recipe Attenuates Airway Inflammation via the TLR4/NF-kB Signaling Pathway on Chronic Obstructive Pulmonary Disease" was published in 2022. Journal: Evid Based Complement Alternat Med.

**Table 2:** The chemical components of Peitu Shengjin Recipe in the negative mode.

NO.	Component name	Area	Retention time	Formula	Precursor mass	Found at mass	Mass error (ppm)	Library score	Isotope ratio difference
1	L(+)-Arginine	8.54*E* + 05	1.3	C_6_H_14_N_4_O_2_	173.104	173.1046	1.0	98.7	1.4
2	Histidine	1.12*E* + 05	1.3	C_6_H_9_N_3_O_2_	154.062	154.0623	0.8	91.7	0.8
3	Aspartic acid	3.76*E* + 05	1.37	C_4_H_7_NO_4_	132.03	132.0304	0.9	88.3	0.6
4	Glutamic acid	7.10*E* + 04	1.38	C_5_H_9_NO_4_	146.046	146.046	0.8	98.2	1.4
5	Sorbitol	2.51*E* + 05	1.42	C_6_H_14_O_6_	181.072	181.0721	1.8	85	0.8
6	D-(+)-Mannose	1.07*E* + 06	1.52	C_6_H_12_O_6_	179.056	179.0563	0.9	80.1	0.6
7	Quinic acid	2.43*E* + 06	1.54	C_7_H_12_O_6_	191.056	191.0563	1.0	89.3	0.5
8	Maltopentaose	9.00*E* + 05	1.59	C_30_H_52_O_26_	827.267	827.2686	1.5	96.1	2.4
9	Maleic acid	7.19*E* + 05	1.63	C_4_H_4_O_4_	115.004	115.0037	0.4	99.6	0.3
10	Citric acid	4.43*E* + 06	2.66	C_6_H_8_O_7_	191.02	191.0201	1.9	99.1	0.6
11	Guanosine	3.39*E* + 05	4.94	C_10_H_13_N_5_O_5_	282.084	282.0848	1.6	99.6	0.2
12	Phenprobamate	1.73*E* + 05	5.77	C_9_H_11_NO_2_	164.072	164.0718	0.9	96.1	0.6
13	Protocatechuic acid	6.14*E* + 04	6.49	C_7_H_6_O_4_	153.019	153.0193	-0.1	93.7	1.8
14	L-Tryptophan	3.43*E* + 05	7.23	C_11_H_12_N_2_O_2_	203.083	203.0828	0.9	97.2	0.5
15	Protocatechuic aldehyde	5.79*E* + 04	7.78	C_7_H_6_O_3_	137.024	137.0245	0.8	96.7	0.9
16	Caffeic acid	1.55*E* + 05	8.61	C_9_H_8_O_4_	179.035	179.035	0.3	91.6	0.7
17	Troxerutin +HCOOH	2.52*E* + 05	9.14	C_33_H_42_O_19_.HCOOH	787.23	787.2313	1.3	99.1	2.4
18	Daidzin	8.91*E* + 04	9.53	C_21_H_20_O_9_	415.103	415.1038	0.8	96.3	2.3
19	p-Coumaric acid	1.03*E* + 05	9.87	C_9_H_8_O_3_	163.04	163.0401	0.5	97.7	1.1
20	Calycosin-7-o-glucoside +HCOOH	1.67*E* + 06	9.96	C_22_H_22_O_10_.HCOOH	491.119	491.1203	1.6	99.6	1.4
21	Neoeriocitrin	4.08*E* + 06	10.12	C_27_H_32_O_15_	595.167	595.1677	1.5	98.6	2.7
22	Liquiritin	1.08*E* + 07	10.19	C_21_H_22_O_9_	417.119	417.1199	1.9	98.8	1.6
23	7-Hydroxycoumarin	5.37*E* + 05	10.33	C_9_H_6_O_3_	161.024	161.0246	1.2	96.6	0.1
24	Isoferulic acid	4.83*E* + 05	10.39	C_10_H_10_O_4_	193.051	193.0508	0.8	98.4	0.5
25	Isochlorogenic acid B	3.49*E* + 05	11.02	C_25_H_24_O_12_	515.119	515.12	1.0	99.8	2.2
26	Apigenin 7-O-beta-D-glucuronide	6.94*E* + 04	11.88	C_21_H_18_O_11_	445.078	445.0779	0.6	88.9	1.7
27	Ononin +HCOOH	1.75*E* + 06	11.99	C_22_H_22_O_9_.HCOOH	475.125	475.1251	1.0	99.5	2.3
28	Methylhesperidin	6.58*E* + 04	12.01	C_29_H_36_O_15_	623.198	623.1988	1.1	89	2.2
29	Platycodin D	6.42*E* + 05	12.43	C_57_H_92_O_28_	1223.57	1223.5716	1.1	92.4	4.5
30	Isoliquiritigenin	9.56*E* + 05	12.49	C_15_H_12_O_4_	255.066	255.0665	1.0	92.7	1
31	Pterostilbene	4.85*E* + 03	12.5	C_16_H_16_O_3_	255.103	255.1027	-0.1	92.7	2.1
32	Eriodictyol	4.30*E* + 04	12.58	C_15_H_12_O_6_	287.056	287.0564	0.9	96.9	2
33	Isomucronulatol-7-O-glucoside	4.20*E* + 05	12.64	C_23_H_28_O_10_	463.161	463.1616	1.4	98.5	1.5
34	Calycosin	8.26*E* + 05	12.7	C_16_H_12_O_5_	283.061	283.0616	1.3	98.9	0.9
35	Xanthotoxol	3.82*E* + 05	12.81	C_11_H_6_O_4_	201.019	201.0196	1.4	91.1	0.7
36	Wogonin 7-O-glucuronide	2.63*E* + 04	13.06	C_22_H_20_O_11_	459.093	459.0937	0.8	97.3	2.3
37	Naringenin	1.33*E* + 06	13.67	C_15_H_12_O_5_	271.061	271.0615	1.2	100	0.8
38	Isorhamnetin	4.21*E* + 04	13.97	C_16_H_12_O_7_	315.051	315.0513	0.9	86.9	1.7
39	Hesperetin	6.93*E* + 05	14.02	C_16_H_14_O_6_	301.072	301.0721	1.0	94.5	2.8
40	Formononetin	7.94*E* + 05	14.72	C_16_H_12_O_4_	267.066	267.0666	1.3	99.2	0.8
41	Pectolinarigenin	1.52*E* + 05	15.18	C_17_H_14_O_6_	313.072	313.072	0.9	98.4	4.5
42	Eupatilin	1.34*E* + 05	15.42	C_18_H_16_O_7_	343.082	343.0827	1.0	92.9	1.5
43	Obacunone	4.44*E* + 04	15.56	C_26_H_30_O_7_	453.192	453.1923	0.9	100	3.8
44	Chrysosplenetin B	5.12*E* + 05	15.59	C_19_H_18_O_8_	373.093	373.0932	0.8	93.9	0.1
45	Astragaloside I +HCOOH	8.18*E* + 05	16.15	C_45_H_72_O_16_.HCOOH	913.48	913.4807	0.5	99.8	2.6
46	Glabridin	4.18*E* + 04	16.78	C_20_H_20_O_4_	323.129	323.1289	-0.1	91.5	0.7
47	Ginsenoside-Ro	2.00*E* + 05	17.18	C_48_H_76_O_19_	955.491	955.4911	0.3	87.9	3.5
48	Gingerglycolipid B +HCOOH	1.30*E* + 05	17.48	C_33_H_58_O_14_.HCOOH	723.381	723.3811	0.4	96.3	1.6
49	Glycyrrhetinic acid	5.68*E* + 04	18.35	C_30_H_46_O_4_	469.332	469.3325	0.3	100	1.4
50	Pachymic acid	1.47*E* + 05	19.46	C_33_H_52_O_5_	527.374	527.3745	0.5	100	0.6

The article "Peitu Shengjin Recipe Attenuates Airway Inflammation via the TLR4/NF-kB Signaling Pathway on Chronic Obstructive Pulmonary Disease" was published in 2022. Journal: Evid Based Complement Alternat Med.

**Table 3:** The pulmonary function assessment in rats with COPD.

Group	FEV0.3/FVC (%)	Cdyn (mL/cmH_2_O)	RI (cmH_2_O/mL/s)
Control	88.96 ± 8.83	0.50 ± 0.06	0.11 ± 0.03
Model	58.64 ± 4.12^▲▲^	0.33 ± 0.04^▲^	0.21 ± 0.03^▲▲^
PSR-low dose	62.94 ± 5.18	0.37 ± 0.04	0.19 ± 0.02
PSR-medium dose	70.04 ± 6.54	0.40 ± 0.05	0.16 ± 0.03
PSR-high dose	72.52 ± 7.02^★^	0.42 ± 0.04^★^	0.12 ± 0.02^★★^
Biostime Probiotic Powder	64.65 ± 6.30	0.41 ± 0.05	0.14 ± 0.02^★^

COPD: chronic obstructive pulmonary disease; Cdyn: dynamic lung compliance; RI: resistance of inspiration; PSR: Peitu Shengjin Recipe. ^▲^*P* < 0.05 and ^▲▲^*P* < 0.01 vs. the control group; ^★^*P* < 0.05 and ^★★^*P* < 0.01 vs. the model group.

**Table 4:** Semiquantitative evaluation of HE in lung tissue of rats with COPD.

Group	Semiquantitative score
Control	−
Model	3.67 ± 0.58
PSR-low dose	3.33 ± 0.58
PSR-medium dose	2.33 ± 0.58^▲^
PSR-high dose	1.67 ± 0.58^▲^
Biostime Probiotic Powder	1.33 ± 0.58^▲▲^

COPD: chronic obstructive pulmonary disease; PSR: Peitu Shengjin Recipe. ^▲^*P* < 0.05 and ^▲▲^*P* < 0.01 vs. the model group.

## Data Availability

All data are available in our study.
